This article has been retracted.

# Atorvastatin Improves Survival in Septic Rats: Effect on Tissue Inflammatory Pathway and on Insulin Signaling

**DOI:** 10.1371/journal.pone.0014232

**Published:** 2010-12-06

**Authors:** Kelly Lima Calisto, Bruno de Melo Carvalho, Eduardo Rochete Ropelle, Francine Cappa Mittestainer, Angélica Costa Aranha Camacho, Dioze Guadagnini, José Barreto Campelo Carvalheira, Mario José Abdalla Saad

**Affiliations:** Department of Internal Medicine, FCM, State University of Campinas (UNICAMP), Campinas, São Paulo, Brazil; University of Las Palmas de Gran Canaria, Spain

## Abstract

The aim of the present study was to investigate whether the survival-improving effect of atorvastatin in sepsis is accompanied by a reduction in tissue activation of inflammatory pathways and, in parallel, an improvement in tissue insulin signaling in rats. Diffuse sepsis was induced by cecal ligation and puncture surgery (CLP) in male Wistar rats. Serum glucose and inflammatory cytokines levels were assessed 24 h after CLP. The effect of atorvastatin on survival of septic animals was investigated in parallel with insulin signaling and its modulators in liver, muscle and adipose tissue. Atorvastatin improves survival in septic rats and this improvement is accompanied by a marked improvement in insulin sensitivity, characterized by an increase in glucose disappearance rate during the insulin tolerance test. Sepsis induced an increase in the expression/activation of TLR4 and its downstream signaling JNK and IKK/NF-κB activation, and blunted insulin-induced insulin signaling in liver, muscle and adipose tissue; atorvastatin reversed all these alterations in parallel with a decrease in circulating levels of TNF-α and IL-6. In summary, this study demonstrates that atorvastatin treatment increased survival, with a significant effect upon insulin sensitivity, improving insulin signaling in peripheral tissues of rats during peritoneal-induced sepsis. The effect of atorvastatin on the suppression of the TLR-dependent inflammatory pathway may play a central role in regulation of insulin signaling and survival in sepsis insult.

## Introduction

Sepsis is one of the most prevalent diseases and one of the main causes of death among hospitalized patients [1]. During the onset of sepsis, the inflammatory system becomes hyperactive, leading to an over-production of pro-inflammatory mediators [2], which contribute to septic shock, multiple organ failure, and death. Hyperglycemia and insulin resistance occur during sepsis, as a consequence of the metabolic effects of stress hormone and cytokine production [3], [4], [5], [6]. Although in the past years there has been considerable progress in our understanding of the pathological pathways that contribute to sepsis and septic shock, pharmacological interventions are currently limited to insulin and activated protein C [7]. Insulin is infused in septic patients with hyperglycemia to normalize glucose levels [7], [8], and it is hypothesized that this reduction in glycaemia is associated with decreased inflammation and endothelial cell damage [4], [5], [6], [9], [10].

Conversely, results from animal studies indicate that insulin may have direct anti-inflammatory effects, independent of its effect on hyperglycemia [11], [12], [13]. However, the mechanism by which insulin reduces inflammation in the absence of hyperglycemia is unknown. Recent data demonstrate that insulin reduces inflammation by activating anti-inflammatory signaling pathways, such as the phosphatidylinositol 3-kinase (PI3K)/protein kinase B (Akt) pathway. Moreover, it is now well established that this pathway negatively regulates LPS-induced signaling and pro-inflammatory cytokine production [14], [15], [16], [17] and activation of PI3K/Akt pathway enhanced survival, whereas inhibition of PI3K reduced survival of endotoxemic mice [15], [18]. In animal models of sepsis, there is a down regulation of the PI3K/Akt pathway that may be the consequence of TLR4 activation and downstream in activation of well established inducers of insulin resistance as JNK, IKK-β and iNOS. Taken together, these data indicate that this insulin signaling pathway, which is reduced in sepsis, may be activated by insulin to mediate the protective effects of insulin in endotoxemia. However, insulin-induced hypoglycemia may counteract the beneficial effects of aggressive insulin therapy in patients with severe sepsis [19].

These data suggest that the ideal drug to improve survival in sepsis should reduce the over-reaction of the inflammatory response and, in parallel, should improve insulin signaling in the PI3K/Akt pathway, without inducing hypoglycemia. Recently, knowledge about statins, a class of powerful hypolipemic drugs with pleiotropic effects, such as anti-inflammatory, antioxidative, immunomodulatory properties, suggest that these agents may offer a novel therapeutic or prophylactic strategy to sepsis [1], [2], [20]. Relevant epidemiological evidence suggests that use of statins may decrease progression to severe sepsis [21], reduce mortality rates [22], [23], [24], [25], [26], [27], [28], [29] and reduce the risk of infections and infection-related complications [30], [31], [32], [33], [34]. However, the mechanisms by which statins induce this protective effect is not well established. The aim of the present study was to investigate whether the ability of atorvastatin to improve survival in sepsis is accompanied by a reduction in tissue activation of inflammatory pathways and, in parallel, an improvement in tissue insulin signaling.

## Results

### Atorvastatin Improves Survival and Protects Against Insulin Resistance in Septic Rats

In the first part of the study, we examined the effect of atorvastatin on the survival curve in animals in which sepsis was induced via CLP. Atorvastatin (10 mg/kg) or placebo was administered by gavage 3 h after surgery or the procedure in sham-operated animals. No deaths occurred in the sham-operated animals, whether or not they had been treated with atorvastatin. The survival curves for rats, in which CLP was performed, are shown in Figure 1A and clearly delineate the benefit sustained from atorvastatin treatment due to improved survival (P<0.0001). As shown in Fig. 1B and 1C, septic animals were more insulin resistant than sham rats; fasting plasma glucose and insulin levels were higher in septic rats than in the control group, and atorvastatin treatment reduced these levels. As depicted by Fig. 1D the plasma glucose disappearance rates measured during the insulin tolerance test (Kitt) were lower in septic animals and atorvastatin treatment reversed these alterations. This improvement is also suggested by the HOMA-IR index, calculated from fasting glycaemia and insulinemia, which is increased in septic animals and significantly decreased in those treated with atorvastatin (Fig. 1E). Atorvastatin treatment had no effect on insulin tolerance in the sham group. Taken together, these data suggest that atorvastatin reversed the sepsis-induced insulin resistance.

**Figure 1:** Effect of atorvastatin on survival in CLP sepsis model. Male Wistars rats, 8 weeks old, were given saline (Sepsis/Sal, n = 20) or atorvastatin 10 mg/kg (Sepsis/Ator, n = 20), 3 h and once a day after CLP. Survival of the rats was monitored at intervals of 12 h for 15 days. The overall difference in survival rate between the groups with and without atorvastatin was significant (P<0.0001) (A). Fasting blood glucose (B). Fasting insulin levels (C). Glucose disappearance rate (D). HOMA-IR index (E). Serum levels of TNF-α (F) and IL-6 (G). Data are presented as means and S.E. of six to eight rats per group. *P<0.05 (Sepsis saline vs. all others groups).

### Effect of Atorvastatin on Serum Levels of IL-6 and TNF-α

The serum levels of IL-6 and TNF-α were also higher in septic animals compared with sham-operated rats. After atorvastatin treatment there was a significant decrease in IL-6 (Fig. 1F) and TNF-α (Fig. 1G) circulating levels.

### Atorvastatin Improves Insulin Signaling in Liver, Muscle and Adipose Tissue of Septic Animals

In the sepsis group, insulin-induced IR and IRS-1 tyrosine phosphorylation were decreased in liver, muscle and adipose tissue when compared with sham rats and these alterations were reversed by atorvastatin (Fig. 2A–F). In parallel, there was a decrease in insulin-induced Akt serine phosphorylation in the liver, muscle and adipose tissue of septic animals when compared with sham rats and atorvastatin was able to reverse these reductions in Akt phosphorylation (Fig. 2G–I). The modulation in IR, IRS-1 and Akt phosphorylation, induced by sepsis and reversed by atorvastatin, was independent of changes in tissue protein expression (Fig. 2A–I). The protein concentration of IR, IRS-1, and Akt did not change between the groups. Equal protein loading in the gels was confirmed by reblotting the membranes with an anti-β-actin antibody (lower panels).

**Figure 2:** Effects of atorvastatin treatment on insulin signaling in the CLP rat. Representative blots show insulin-induced tyrosine phosphorylation of Insulin Receptor β (IRβ) in liver (A), muscle (B) and adipose (C) of sham and septic rats. Total protein expression of IRβ (A–C, lower panels). Insulin-induced tyrosine phosphorylation of Insulin Receptor Substrate 1 (IRS1) in liver (D), muscle (E) and adipose tissue (F) of sham and septic rats. Total protein expression of IRS1 (D–F, lower panels). Insulin-induced serine phosphorylation of Akt in liver (G), muscle (H) and adipose (I) of sham and septic rats. Insulin-induced threonine phosphorylation and total protein expression of Akt (G–I, lower panels). In this case, blots were stripped and reprobed with β-actin (A–I, lower panels) to confirm equal loading of proteins. Data are presented as means +/− S.E.M from 6–8 rats per group. *P<0.05 (Sepsis/Sal vs. all others groups). IB, immunoblot; CLT: Sham/Saline; ShT: Sham/Atorvastatin; SAL: saline; ATOR: atorvastatin.

### Atorvastatin Attenuates Sepsis-Induced Inflammatory Changes

Toll-like receptor 4 (TLR4) is a transmembrane receptor that participates in pathogen recognition during the inflammatory response, and leads to cytokine and other immune-related gene expression [35], [36]. During sepsis, the activation of TLR4 signaling induces upregulation of intracellular inflammatory pathways, such as the IκB kinase β (IKK-β)/nuclear factor kappa B (NFκ-B) pathway.

Next, we examined the immunomodulatory effects of atorvastatin on TLR4 activation in liver, muscle and adipose tissue of septic animals. Fig. 3 shows that sepsis induced TLR4 protein levels and activation, as demonstrated by an increase in TLR4/MyD88 interaction in the three tissues investigated, and atorvastatin reduced this early step of TLR4 activation and also TLR4 expression (Fig. 3A–C).

**Figure 3:** To evaluate the association of TLR4 with MyD88, immunoprecipitations were performed with MyD88 antibody followed by immunoblotting with TLR4 specific antibody. Representative blots show TLR4 activation (upper panels) and expression (lower panels) in liver (A), muscle (B) and adipose tissue (C) of sham and septic rats. IKKβ phosphorylation in liver (D), muscle (E) and adipose (F) of sham and septic rats. Total protein expression of IKKβ (D–F, lower panels). Phosphorylation of IκBα in liver (G), muscle (H) and adipose (I) of sham and septic rats. Data are presented as means ±S.E.M from 6–8 rats per group. *P<0.05 (Sepsis/Sal vs. all other groups); **P<0.001 (Sepsis/Sal vs. control); #P<0.05 (Sepsis/Sal vs. Sepsis/Ator). IB, immunoblot; CLT: Sham/Saline; ShT: Sham/Atorvastatin; SAL: saline; ATOR: atorvastatin.

Downstream of TLR4 activation, we examined the IKK–NF-κB pathway, an important regulator of inflammation and insulin resistance. The main function of the IKK complex is the activation of NFκB through phosphorylation and degradation of IκBα [37], [38]. NFκB activity was monitored using IKKβ and IκBα phosphorylation, as described previously [39]. As expected, IKKβ and IκBα phosphorylation were increased in liver, muscle and adipose tissue of septic animals and atorvastatin decreased these phosphorylations in the tissues investigated (Fig. 3D–I).

JNK activation was determined by monitoring phosphorylation of JNK (Thr183 and Tyr185) and c-Jun (Ser63), which is a substrate of JNK. JNK phosphorylation in liver, muscle and adipose tissue were increased in septic animals and atorvastatin induced a downmodulation in the phosphorylation of this serine kinase (Fig. 4A–C). Consistent with JNK activation, c-Jun phosphorylation was induced by sepsis and reversed by atorvastatin in the tissues investigated (Fig. 4D–F).

**Figure 4:** Representative blots show the JNK phosphorylation in liver (A), muscle (B) and adipose tissue (C) of sham and septic rats (upper panels). Total protein expression of JNK (A–C, lower panels). Phosphorylation of c-jun in liver (D), muscle (E) and adipose tissue (F) of sham and septic rats. Serine 307 Phosphorylation of IRS1 in liver (G), muscle (H) and adipose tissue (I) of sham and septic rats (upper panels). Total protein expression of IRS-1 (G–I, lower panels). Data are presented as means ± S.E.M from 6–8 rats per group. *P<0.05 (Sepsis/Sal vs. all others groups); **P<0.001 (Sepsis/Sal vs. control); #P<0.05 (Sepsis/Sal vs. Sepsis/Ator). IB, immunoblot; CLT: Sham/Saline; ShT: Sham/Atorvastatin; SAL: saline; ATOR: atorvastatin.

We also investigated Ser307 phosphorylation of IRS-1 in liver, muscle, and adipose tissue in the four groups of rats. Ser307 phosphorylation was induced by sepsis in the three tissues and the treatment with atorvastatin reversed this alteration (Fig. 4G–I). NFκB nuclear subunit p50 expression was determined in nuclear extracts and we found an increase in this subunit in nuclear extracts of septic animals, but there was a clear decrease in the three tissues after atorvastatin treatment (Fig. 5A–C). The tissue expressions of iNOS (Fig. 5D–F) and IL-6 (Fig. 5G–I) were higher in liver, muscle and adipose tissue of septic rats that received saline, and were significantly reduced by atorvastatin treatment.

**Figure 5:** Representative blots show the NFkB activation in nuclear fractions of liver (A), muscle (B) and adipose tissue (C) of sham and septic rats. In this case blots were stripped and reprobed with actin (A–C, lower panels) to confirm equal loading of proteins. Tissue levels of iNOS (D–F) and IL-6 (G–I) expression in liver, muscle and adipose tissue of sham and septic rats. Data are presented as means ± S.E.M from 6–8 rats per group. *P<0.05 (Sepsis/Sal vs. all others groups); **P<0.001 (Sepsis/Sal vs. control); #P<0.05 (Sepsis/Sal vs. Sepsis/Ator). IB, immunoblot; CLT: Sham/Saline; ShT: Sham/Atorvastatin; SAL: saline; ATOR: atorvastatin.

Previous studies have shown that sepsis is also characterized by endoplasmic reticulum stress. It is clear that ER stress can also induce activation of JNK and IKKβ. We then investigated the effect of sepsis (treated or not with atorvastatin) on proteins that reflect ER stress. Our data showed that sepsis induced ER-stress, as determined by the increased phosphorylation of the ER membrane kinase, PERK (PKR-like endoplasmic reticulum kinase) and its substrate (Fig. 6A–C), eIF2α (eukaryotic translation initiation factor 2α) (Fig. 6D–F) and increased the expression of ATF6α (Fig. 6G–I). Treatment with atorvastatin significantly reduced the expression of all markers of ER-stress. (Fig. 6A and D)

**Figure 6:** Representative blots show the PERK phosphorylation in liver (A), muscle (B) and adipose tissue (C) of sham and septic rats. eIF2α phosphorylation (D–F) and ATF6 (G–I) expression in liver, muscle and adipose tissue of sham and septic rats. In this case, blots were stripped and reprobed with actin (A–I, lower panels) to confirm equal loading of proteins. Data are presented as means ± S.E.M from 6–8 rats per group. *P<0.05 (Sepsis/Sal vs. all others groups); #P<0.05 (Sepsis/Sal vs. Sepsis/Ator). IB, immunoblot; CLT: Sham/Saline; ShT: Sham/Atorvastatin; SAL: saline; ATOR: atorvastatin.

## Discussion

In sepsis, the acute immune response is organized and executed by innate immunity. This response starts with sensing of danger by pattern-recognition receptors on the immune competent cells and endothelium. The pattern-recognition receptors, mainly toll-like receptor (TLR), are also activated in other tissues such as liver, muscle and adipose tissue [40]. The sensed danger signals, through specific signaling pathways, activate transcription factors and gene regulatory systems, which up-regulate the expression of pro-inflammatory mediators. However, the over-reaction of this pro-inflammatory response has an important role in the development of multiple organ failure and death. The combinations of the activation of pattern recognition receptors, specifically TLR4, and the cytokine storm of sepsis have an important role in insulin resistance. In this regard, tissue insulin resistance may be used as an important indicator of the resultant actions of pattern recognition receptors and the induction of the pro-inflammatory cytokines, being a tissue marker of severity of sepsis, before organ failure. In addition, this insulin resistance may also aggravate sepsis, as previously described [3], [4], [41]. In this regard, we believe that the evaluation of insulin signaling pathway through PI3K/Akt in liver, muscle and adipose tissue may be important indicators of this over-reaction at the tissue level, and the improvement in this signaling pathway, induced by some treatments, in parallel with a decrease in tissue inflammation, may predict the effectiveness of this treatment.

In the present study, we demonstrated that atorvastatin improves survival in septic rats, decreases circulating inflammatory cytokines and improves insulin resistance, in parallel with a decrease in TLR4 signaling and an improvement in insulin signaling in liver, muscle and adipose tissue. The improvement in survival of septic animals when using statins has been previously described, and was related to a complete preservation of cardiac function and hemodynamic status and also a reversion of increased monocyte adhesion to the endothelium, all of which were altered in septic animals without treatment [42], [43].

Our data show that atorvastatin, administered 3 hours after the induction of sepsis, is able to improve the survival curve, attenuating higher levels of IL-6 and TNF-α and reduce insulin resistance, as demonstrated during the insulin tolerance test. In septic animals, insulin resistance was accompanied by a reduction in insulin-induced IR, IRS-1 tyrosine phosphorylation and in insulin-induced Akt phosphorylation, in liver, muscle and adipose tissue. Since Akt has a critical role in protection from apoptosis, it is possible that the reduced insulin signaling through this IRSs/PI3K/Akt pathway, in sepsis, may contribute to multi-organ failure by preventing or delaying apoptosis [14], [15], [44]. In this study, we demonstrate that pretreatment with atorvastatin inhibits sepsis-induced insulin resistance by improving insulin signaling via the IR–IRS-1–Akt pathway in target tissues. This restoration of insulin signaling in these tissues would allow the animal to have an appropriate control of hepatic glucose output and of the peripheral glucose uptake and storage. In addition, skeletal muscle and adipose tissue contribute to IL-6 expression during sepsis [45], [46], [47], and since the anti-inflammatory effect of insulin is mediated through the PI3K pathway [14], [15], [18], we can speculate that the restoration of this pathway in the insulin-dependent tissues, induced by atorvastatin in septic animals, may have also contributed to the anti-inflammatory effect of this drug.

During the past ten years, accumulating evidence shows a clear molecular interaction between metabolic and immune signaling systems in different situations of insulin resistance [40], [48], [49]. We and others have previously demonstrated that TLR4 signaling is activated in diet induced obesity (DIO), and that this activation culminates in an increase in the activation of downstream effectors such as IKKβ, JNK and iNOS, which have critical roles in insulin resistance [40]. In septic animals, there was an increase in TLR4 activation and also in downstream effectors that may have an important role in the insulin resistance of these animals [50]. Our data show that atorvastatin decreases TLR4 expression/activation, a modulation that might have a role in the attenuated expression of inflammatory mediators in response to a septic insult. The reduction in TLR4 expression/activation, observed in our study, is in accordance with a previous study that also observed this effect on TLR4 expression/activation with different statins and cell types [51].

The immune modulator activity of atorvastatin was evident downstream from TLR4, at the level of IKK/IκB/NF-κB pathway activation. Atorvastatin induced a significant decrease in IKK phosphorylation and, as expected, an increase in IκB phosphorylation, suggesting a deactivation of this pathway. NF-κB has been documented to play a major role in sepsis induced inflammatory cytokine expression [52], [53], [54]. Our findings suggest that NF-κB, which is normally translocated from the cytoplasm to the nucleus after sepsis insult, was strongly inhibited by atorvastatin in the three target tissues studied. This result suggests that the atorvastatin-mediated inhibition of cytokine production may be the consequence of the modulation of the IKK/IκB/NF-κB pathway by this drug.

The activation of NF-κB with its translocation to the nucleus is able to induce the increase in TNF-α, IL-6 and in iNOS in septic animals [37], [38], [55]. TNF-α is one of the crucial pro-inflammatory cytokines; however, when over produced by deregulation or persistent infection, TNF-α may induce septic shock and contributes to insulin resistance, and its levels are drastically elevated in a number of forms of human sepsis, in turn correlating with increased mortality [56]. Specifically, iNOS and IL-6 have been shown to be produced early in the response and have been suggested to play critical roles in driving physiological/pathological responses that lead to septic shock [57]. We further investigated the effects of atorvastatin on the production of these inflammatory proteins in tissues and serum of septic rats. In accordance with previous data, atorvastatin treatment inhibited iNOS, TNF-α and IL-6 expression in the muscle, liver and adipose tissues of septic rats, and also the circulating levels of TNF-α and IL-6. [58]. Previous studies have demonstrated that skeletal muscle and adipose tissue contribute to IL-6 production during endotoxemia [45], [46], [47], and the anti-inflammatory effects of atorvastatin on IL-6 production in sepsis may be the result of the direct activation of PI3K pathway in these tissues. The atorvastatin-mediated reduction of these negative modulators of insulin signaling may have an important role in the improvement of insulin signaling observed in the three tissues of septic animals.

Another TLR4 downstream pathway by which atorvastatin could attenuate the inflammatory response induced by sepsis is through JNK, a serine kinase that is responsible for activation of the inflammatory pathway by phosphorylation of the c-Jun and ATF2 transcription factors [59], [60]. Several studies suggest that JNK contributes to insulin resistance by phosphorylating IRS-1 at serine 307, and this phosphorylation leads to inhibition of IRS-1 function [26], [27], [30], [33], [61], [62], [63], [64], although this has very recently been questioned [65]. Here, we observed that sepsis led to serine phosphorylation of IRS-1 and that atorvastatin reversed this phenomenon in three target tissues, in parallel with a reduction in JNK activity. Our data showing that atorvastatin inhibits JNK phosphorylation/activation in septic rats indicate that the beneficial effect of this drug in improving survival and reducing insulin resistance is mediated by different pathways.

Besides being activated by TLR4, JNK activity is induced in different pathophysiological states including infection, inflammation, obesity and hyperlipidemia, also as a consequence of ER stress [66], [67], [68]. The cellular response to ER stress, referred to as UPR, results in the activation of three linked signal transduction pathways emanating from three principle ER stress sensors: IRE1α, double-stranded RNA–dependent protein kinase–like kinase (PERK) and ATF6α [49], [69]. Mechanistically, activation of the UPR contributes to the decrease in insulin sensitivity through IRE1α-dependent activation of c-Jun N-terminal kinase (JNK) [70], [71]. Recently, it was demonstrated that statins are able to prevent ER stress [72]. In the present study, we confirm this finding by showing that atorvastatin strongly inhibited phosphorylation of IRE1α and PERK and ATF6α expression, suggesting that this drug can attenuate the ER-stress induced by sepsis.

Overall, our data demonstrate that atorvastatin exerts direct regulatory effects on TLR4 expression/activation in an animal model of sepsis that influences TLR4 signaling. Atorvastatin reduces TLR4 surface expression on liver, muscle and adipode tissues, causing downregulation of proinflammatory pathways such as IKK and JNK, leading to a decrease in NF-κB activation and cytokine expression. In addition, atorvastatin also decreases ER stress and, consequently, the activation of JNK and IKK. Thus, we suggest that the effects of atorvastatin on TLR4 expression/activation and on ER stress are mechanistically relevant to improve the sepsis-induced insulin resistance. There are several potential limitations to the present study.

To date, pharmacological interventions in sepsis have usually been limited to insulin and Protein C [7]. The beneficial effects of activated protein C are partially independent from its anticoagulant activity and may be related to anti-inflammatory and anti-apoptotic effects, but its effect on insulin signaling is unknown. Insulin has anti-inflammatory effects [11], [12], [13], [19], which are dependent on PI3K signaling, and the infusion of this hormone induces the PI3K/Akt pathway. However, the beneficial effect of insulin may be overcome by hypoglycemia. It is important to mention that, in sepsis, many inflammatory pathways are activated in parallel with a reduction in the PI3K/Akt pathway, thus, merely blocking a single component of the inflammatory pathways or inducing the activation of PI3K may be insufficient to arrest the process. In this regard, our data show that atorvastatin is able to modulate entire families of inflammatory mediators, associated with a clear improvement in tissue insulin signaling and in insulin sensitivity, suggesting mechanisms for its efficiency in sepsis. Additionally, our data may suggest that the investigation of drugs in sepsis should take into account tissue measurements of inflammatory pathways and insulin signaling, or other early tissue markers that indicate the severity of sepsis.

In summary, this study demonstrated that treatment with atorvastatin increased survival with a significant effect upon insulin sensitivity, improving insulin signaling in peripheral tissues of the rat during peritoneal-induced sepsis. This drug reduces TLR4 activation, in association with downstream JNK and IKK/NF-κB activation and downregulated the serum levels of cytokine release. The effect of atorvastatin on TLR-dependent inflammatory pathway suppression may play a central role in the regulation of insulin signaling and survival following the sepsis insult.

## Materials and Methods

### Materials

Anti-IR-β (α-IR), anti-IRS-1, anti-Akt, anti-p-JNK, anti-iNOS, anti-NFκB, anti-IL6, anti-TLR4, anti-IKKβ, anti-pIKKβ, anti-pIκBα, anti-MyD88, anti-p-cjun, anti-pJNK, anti-pPERK anti-PERK, anti-ATF6α and anti-IRE1α antibodies were from Santa Cruz Technology (Santa Cruz, CA, USA). Anti-pAkt was from Cell Signaling Technology (Beverly, MA, USA). Anti-phospho-IRS-1^ser307^ was obtained from Upstate Biotechnology, Inc. (Lake Placid, NY, USA). Anti-peIF2α was from Abcam (Cambridge, MA, USA). Atorvastatin was obtained from Pfizer (Loughbeg, County Cork, Ireland). Human recombinant insulin was from Eli Lilly and Co. (Indianapolis, Indiana, USA). Routine reagents were purchased from Sigma Chemical Co. (St. Louis, MO, USA), unless specified elsewhere.

### Animal Care and Experimental Procedures

All experiments were approved by the Ethics Committee at the University of Campinas, CEEA/Unicamp 1267-1. Male Wistar- Hannover (8 wks old) were maintained in a room with 12-hour day/night cycles and room temperature of 21°C, with food and water *ad libitum*. Wistar rats were randomly divided into four groups; atorvastatin-treated sepsis (Sepsis/Ator), saline-treated sepsis (Sepsis/Sal), atorvastatin-treated sham (Sham), and saline-treated sham (Control).

Cecal ligation and puncture (CLP) was performed, as previously described [73], and is a commonly-used surgical technique in rodents and thought to be a clinically relevant animal model of sepsis. Anesthesia was induced by IP administration of ketamine (80 mg/kg BW) and xylazine (15 mg/kg). Through a 1-cm abdominal midline incision, the cecum was ligated below the ileocecal valve with careful attention to avoid obstruction of the ileum or colon. The cecum was subjected to a four “through-and-through” perforations (20-gauge needle). The abdominal incision was closed in layers. Sham-operated rat underwent the same procedure, except for ligation and perforation of the cecum. All procedures were performed under sterile conditions. Animals were allowed to recover and were observed twice a day. Three hours after the induction of sepsis and every 24 hours rats received atorvastatin (10 mg/kg) or an equivalent volume of saline by oral gavage. The dose of atorvastatin was chosen on the basis of previous findings [74] and was consistent with the maximum human dose (1.1 mg/kg per day), and the higher metabolic rate of the drug in rodents [75].

### Homeostasis Model Assessment

Insulin resistance was assessed from fasting insulin and glucose levels, using the previously validated homeostasis model of assessment (HOMA-IR), as previously described [76], [77]. HOMA-IR was calculated by the formula: fasting plasma glucose (mmol/l) x fasting plasma insulin (mU/l)/22.5. Fasting blood glucose was measured by the glucose oxidase method. Plasma insulin was assayed using commercial rat-specific radioimmunoassay kits (Linco Research Inc, St. Louis, MO, USA).

### Insulin tolerance Test (ITT)

The insulin tolerance test (ITT) was performed on these rats at 24 hours after sepsis, as previously described [78]. Insulin (1.5 U/kg) was administered by i.p. injection and blood samples were collected at 0, 5, 10, 15, 20, 25, and 30 min to determine serum glucose. The constant rate for glucose disappearance (Kitt) was calculated using the formula 0.693/t1/2. Glucose t1/2 was calculated from the slope of the least-squares analysis of plasma glucose concentrations during the linear decay phase [76].

### Cytokines Assays

IL-6 and TNF-α were determined using commercially available ELISA kits (Pierce Biotechnology Inc., Rockford, IL, USA), following the instructions of the manufacturer.

### Tissue Extraction, Immunoprecipitation and Immunoblotting

Rats were anaesthetized by intraperitoneal injection of sodium thiopental and were used 10–15 min later, *i.e.* as soon as anesthesia was assured by the loss of pedal and corneal reflexes. Five minutes after saline (0.2 ml) or insulin injection (3.8 U/Kg ip), liver, muscle and adipose tissue were removed, minced coarsely and homogenized immediately in extraction buffer, as described elsewhere. Extracts were used for immunoprecipitation with MyD88 and Protein A-Sepharose 6MB (Pharmacia, Uppsala, Sweden). NFκB p50 activation was determined in nuclear extracts from liver, muscle and adipose tissue, as previously described [79]. The precipitated proteins and/or whole tissue extracts were subjected to SDS-PAGE and immunoblotting, as previously described [40], [78].

### Statistical Analysis

The overall difference in survival rate was determined by the Kaplan–Meier test followed by log–rank test. Specific protein bands present in the blots were quantified by digital densitometry (ScionCorp Inc., Frederick, MD, USA). Means ± S.E.M. obtained from densitometric scans, area measurements, and the values for blood IL-6, TNF-α and glucose were compared by ANOVA with post hoc test (Bonferroni). A P value of *p*<0.05 was accepted as statistically significant.
